The article "Strategies for Oxygen Ecosystems in Middle-Income Countries: A Review and Case Study from Lebanon" was published in 2024. Journal: Emerg Med Int.

# Strategies for Oxygen Ecosystems in Middle-Income Countries: A Review and Case Study from Lebanon

**DOI:** 10.1155/2024/9964636

**Published:** 2024-02-02

**Authors:** Tim Baker, Claudio Gatti, Guido Rossini, Habtamu Tolla, Anne Detjen, Mulugeta Mideksa, Nadeen Hilal, Rima Shaya

**Affiliations:** ^1^Queen Mary University of London, London, UK; ^2^Department of Global Public Health, Karolinska Institutet, Stockholm, Sweden; ^3^Department of Emergency Medicine, Muhimbili University of Health and Allied Sciences, Dar es Salaam, Tanzania; ^4^Think Global Srl, Rome, Italy; ^5^UNICEF Headquarters, New York, USA; ^6^UNICEF Middle East and North Africa, Amman, Jordan; ^7^Ministry of Public Health, Government of Lebanon, Baabda, Lebanon; ^8^UNICEF Lebanon Country Office, Beirut, Lebanon

## Abstract

The COVID-19 pandemic led to a surge of critically ill patients and a sudden increase in the need for oxygen treatment worldwide. Pre-existing gaps in oxygen systems became apparent, and governments, multilateral agencies, and other partners scrambled to increase the production, supply, and use of oxygen to meet this need. The importance of an oxygen ecosystem that is appropriate for the local context became clear. This review describes strategies for oxygen ecosystems in middle-income countries, with specific experiences from Lebanon, following the authors' extensive assessment of the country's oxygen ecosystem, on behalf of the government and UNICEF. In the assessment, fifteen governmental hospitals were visited and evaluated using the UNICEF Oxygen System Planning Tool, discussions were held with key stakeholders, and documents were reviewed. An optimal oxygen ecosystem needs to take into consideration the production of oxygen and delivery to facilities, the maintenance system within facilities, and the clinical use of oxygen. Lebanon, a lower-middle income country in the Middle East, is contending with an extensive economic crisis affecting the health system. Eighteen recommendations for strengthening the oxygen ecosystem in Lebanon that are relevant for other middle-income countries include the establishment of a National Oxygen Committee, installation of additional oxygen plants, strengthened systems for maintenance and electricity supply, increased production, procurement and supply chain resilience, improved training and human resources, the use of data collection and regular information to guide the ecosystem, and integration of oxygen into the rest of the health system.

## 1. Background

Oxygen is a requirement for life. In ill-health and particularly in severe forms of ill-health—“critical illness”—patients can develop low levels of oxygen in their bodies. Just one disease, pneumonia, causes critical illness with low oxygen levels in an estimated 7 million children in low- and middle-income countries each year [1]. To improve outcomes for critically ill patients, it is standard practice to provide patients with oxygen. Without oxygen therapy, many critically ill patients would die. Oxygen is used for a wide range of medical conditions: childhood and adult pneumonia, infectious diseases, noncommunicable diseases, injuries, maternal haemorrhage and eclampsia, and in surgery, anaesthesia, and intensive care. Oxygen is an essential medicine, and the ability to identify when it is needed [2–4] and to provide it to all who need it are crucial functions of all health systems [5–8].

The COVID-19 pandemic led to a surge in the number of critically ill patients and a sudden increase in the need for oxygen treatment worldwide. Governments, multilateral agencies, and other partners scrambled to increase the production, supply, and use of oxygen to meet this need [8]. In many settings, the need outstripped the supply, leading to substantially increased morbidity and mortality. It has become clear that a high-quality oxygen ecosystem requires the integration of many diverse components [9]. The pandemic highlighted how all countries require such an ecosystem to be robust and context-appropriate both for the general health needs of their populations and to be prepared for critical illness surges in public health emergencies [10].

The optimal oxygen ecosystem depends on the local context. High-income countries have developed resource-intensive ecosystems, with substantial primary systems and extensive backup plans in case of system failures [11]. For middle-income countries, resources are more constrained, and the limited resources need to be carefully managed to produce the greatest health impact [12]. In such settings, the optimal oxygen ecosystem has not been well described, taking into account competing health priorities and global demands. This review aims to use the literature to describe strategies for oxygen ecosystems in middle-income countries. A systematic review of the literature was not conducted. Each section of the review contains specific experiences from Lebanon following the authors' extensive assessment of the country's oxygen ecosystem conducted on behalf of the government and UNICEF in 2022-2023. In the assessment, fifteen governmental hospitals were visited, and their oxygen systems were evaluated using the UNICEF Oxygen System Planning Tool [13]; discussions were held with key stakeholders, and documents were reviewed.

*Lebanon, on the eastern side of the Mediterranean Sea, has a population of 7 million people and is a lower-middle income country with a gross domestic product (GDP) per capita of $4,500USD. Life expectancy is 76.4 years, under 5, mortality is 7 per 1,000 live births, and the maternal mortality ratio is 29 per 100,000 live births [14]. In the past few years, Lebanon has contended with several crises, an economic crisis, the COVID-19 pandemic and an explosion in the Port of Beirut. Since 2018, Lebanon's economic output has halved, inflation is over 100%, and the average food basket price has increased six-fold [15]. Unemployment is high, and poverty is increasing. There are acute shortages of fuel and electricity blackouts and large challenges for the health system including supply shortages [16]. The waves of COVID-19 in the country have led to over 1.2 million confirmed cases and 10,000 deaths. The Port of Beirut explosion in 2020 led to over 200 deaths, 7000 injuries, and damage of approximately $4 billion.*

## 2. Oxygen Production and Delivery to Facilities

All countries require oxygen, either produced in country or imported from abroad. The amount of oxygen to cover both basic and surge needs has been the topic of accelerated work in the last few years, stimulated by the COVID-19 pandemic. Tools produced by WHO and UNICEF [17, 18] and others [19] have been introduced, and extensive research is ongoing to provide robust estimates of the need through initiatives such as the Lancet Commission on Oxygen Security [20].

Oxygen for medical use must be free of contaminants and can be produced through different technologies. Liquid oxygen (LOX) plants separate oxygen from nitrogen and other gases using very cold temperatures, high pressure, and distillation (cryogenic distillation), producing oxygen in liquid form. They are usually commercial factories and may be producing gases primarily for other industries. To distribute oxygen, cylinders are filled with gaseous oxygen at the factory and transported to health facilities, or liquid oxygen is transported to facilities and kept in on-site tanks and converted to gaseous oxygen when required. Pressure swing adsorption (PSA) plants separate out oxygen by compressing air through a specialised adsorbent material. Vacuum swing adsorption (VSA) plants are a newer technology that use a vacuum rather than a compressor [21]. PSA plants are often located at health facilities, and the oxygen provided to hospital wards through piping, or a compressor at the plant can fill cylinders for transportation. There are relative advantages and disadvantages of LOX and PSA (Figure 1). Oxygen can also be produced by small, bedside oxygen concentrators that use similar technology to PSA plants to provide low-flow oxygen directly to patients, either for home-use, or in health facilities, especially at lower levels of care where high-flow rates are not required.

While comparisons have found that the cost of oxygen production is similar in LOX and PSA plants, PSA oxygen may be cheaper per unit delivered to the patient, due to the additional supply and transportation costs of LOX [22]. The cost of oxygen is impacted by the relationship between plant capacity and oxygen demand—with the greatest efficiency when the capacity of a plant is similar to the demand [23].

LOX plants produce oxygen at a concentration of approximately 99%. PSA plants produce oxygen at a concentration of approximately 93%. The first global standards for medical oxygen covered only LOX, specifying a minimum oxygen content of 99%. With the expansion of PSA plants, standards have been updated to include an oxygen concentration of 90%–96%. The European Pharmacopoeia includes two monographs on oxygen: oxygen (0417) and oxygen (93%) (2455), and the United States Pharmacopoeia includes oxygen 93%. In 2021, WHO included oxygen 93% in the draft of the 11^th^ edition of the International Pharmacopoeia. The International Organization for Standardization standards for medical gas pipeline systems include 93% oxygen, and the WHO has stated that medical oxygen must have a concentration above 82% [17]. For the majority of patients treated with oxygen who are provided with a mix of air and oxygen, there is no clinical difference between 99% and 93% oxygen. For a few special patient groups, there has been debate as to whether provision of 99% rather than 93% has a meaningful clinical impact. While evidence is scarce, there are important rationales [24] and increasing calls to promote 93% or 99% as clinically equivalent in order to increase oxygen access [25].

*Prior to the COVID-19 pandemic, oxygen was not reported to be in short supply in Lebanon. Most oxygen was supplied to hospitals as LOX by a duopoly of private suppliers and stored in on-site tanks. Primary healthcare facilities rarely had oxygen and referred patients to hospital if they required oxygen. There were four PSA plants in public hospitals in the country. During the pandemic, oxygen demand increased five-to-ten-fold, due to the surge in critically ill patients along with the increased use of high-flow oxygen and mechanical ventilation. The private suppliers increased their supply to hospitals, refilling tanks every day in some hospitals (personal communication). The number of intensive care beds in public hospitals tripled—from 300 beds for COVID in August 2020 to 1176 by April 2021, of which 90% were occupied [26]. However, there were concerns regarding quality of care including oxygen therapy for critically ill COVID-19 patients as skilled staff and systematic implementation of care protocols were lacking [26]. As in many countries, there were sporadic reports of acute shortages of oxygen supply [27] and access [27]. As LOX had been so dominant in Lebanon, there had not previously been demand for other forms of oxygen production, and some clinicians reported concerns about the quality of non-LOX oxygen (personal communication).*

## 3. Oxygen Engineering, Maintenance in Facilities, and Electricity Supply

Once oxygen is within a health facility, a reliable delivery system is needed. First, oxygen is stored in a safe and secure way in the form of compressed gas cylinders, liquid oxygen tanks, or on-site generation systems. From this source, a network of pipes distributes oxygen to wall outlets by patient beds and other points of use throughout the hospital. Oxygen cylinders can also be filled at the source and transported within the hospital. The oxygen system requires pressure regulators, safety valves, and alarms to ensure oxygen is delivered safely. At the patient, flow meters allow health workers to accurately control oxygen delivery.

Maintenance of oxygen systems is crucial to ensure the safe and efficient operation of the system and to prevent failures that could be life-threatening. The system should be cleaned and inspected regularly and tested for leaks. The flow meters should be calibrated regularly, the concentration and purity of the oxygen should be accurately checked, and preventive maintenance should be conducted, so worn or damaged parts can be replaced early. Facilities require biomedical engineers or technicians with expertise to maintain the oxygen system, with regular training on maintenance and repairs, and the hazards associated with oxygen systems. Specialist engineers may be needed for facilities with in-house oxygen generation or complex systems.

Health facilities require backup systems to ensure a continuous supply of oxygen in case of a primary system failure. This can involve reserve tanks of compressed oxygen, backup generators to ensure a continuous supply of electricity, portable oxygen tanks of compressed oxygen in case of a failure in the primary piping system, and cylinder changeover systems (manifolds) that automatically switch between banks of cylinder. Health facilities must have regularly tested emergency plans to ensure that patients continue to receive the oxygen they need in case of primary system failure.

Oxygen production and use require a large supply of electricity and a supply that is reliable and constant. Power outages or failures can have a catastrophic impact on oxygen production and delivery. It should be stated however that hospitals are electricity-intensive facilities, and the oxygen ecosystem accounts for only a small proportion of the total energy need.

*In Lebanon, all the 15 assessed hospitals had a centralised distribution system for oxygen and other medical gases, with backup systems composed of one or more cylinder changeover systems. Hospitals had technicians with expertise to manage medical oxygen; however, training levels were variable, and refresher training had not been held for some time. In some hospitals, the distribution system was in need of important maintenance. The energy supply in Lebanon has significant challenges, with the national grid providing energy for only a few hours each day. Electricity supply in hospitals and throughout the country is dependent on on-site diesel generators, risking power shortages. All medical equipment including oxygen has been estimated to use 14% of energy in Lebanese public hospitals* [28].

## 4. Clinical Use of Oxygen

For most patients, oxygen is provided through nasal prongs (small plastic tubes in the nostrils) or face masks (plastic mask covering the mouth and nose). Patients who require higher concentrations can be provided with a mask with a reservoir bag. The patient breathes a mixture of oxygen from the oxygen source and room air from around the sides of the prongs or mask. The flow of oxygen is usually between 0.5 litres and 6 litres per minute and can be increased up to 15 or 20 litres per minute. The concentration of the oxygen in the gas mixture that they breathe varies between 21% and approximately 80% and can be modified by the clinician through adjusting the oxygen flow rate and the choice of the type of prongs or mask.

Some severely ill patients require higher concentrations, flows, or pressures of oxygen and receive oxygen via a noninvasive ventilation mask that is firmly attached over the nose and mouth. This prevents room air from leaking in and allows oxygen to be delivered under pressure. High-flow nasal oxygen can also be provided using specialised equipment with oxygen-air mixtures of up to 60 litres per minute.

A minority of critically ill patients are intubated—a tube is inserted into the trachea through which oxygen can be provided. Room air cannot leak in, and the gas mixture is decided by the clinician using an oxygen source and a source of air (usually compressed)—usually between 30% and 50% oxygen and sometimes up to 80% or 90% oxygen—and the patient has their breathing assisted with mechanical ventilation.

The clinical use of oxygen requires a sustainable source of supplies and staff with expertise to treat patients with oxygen. Staff should receive regular training on the indications for oxygen therapy and its safe and effective use. Specialist staff may be needed for facilities that provide advanced oxygen therapy such as high-flow nasal oxygen, intubation, and mechanical ventilation.

Oxygen is a medicine and should be used rationally. Undertreatment of hypoxia is a large clinical problem globally. Overtreatment is also a problem, with high-flow rates of oxygen being used when not needed, and oxygen therapy continuing beyond the point when the patient has recovered, risking hyperoxia and side effects in newborns and other patient groups [29].

Patients who require oxygen therapy are critically ill. They have a life-threatening condition and often require other care beyond oxygen therapy. The first line, most basic care required by critically ill patients has recently been defined as essential emergency and critical care [30], and 40 clinical processes have been specified including oxygen therapy, intravenous fluids, and patient positioning to maintain a free airway. Ensuring systems are in place, staff trained and that this care is provided to all critically ill patients including those who require oxygen is crucial for all hospitals in all settings [31].

*The Lebanese Ministry of Public Health (MOPH) oversees the health system in the country. For many years, Lebanon has had a well-functioning health system [32] and has ranked 33rd among 195 countries in the Healthcare Access and Quality index [33]. The MOPH runs a network of primary healthcare centres and dispensaries without in-patient services. There is a large private healthcare delivery system in the country, and public facilities account for only 18% of in-patient hospital beds—there are 127 private and 32 public hospitals [33]. The ongoing crises in the country have severely affected the health system. Public hospitals have struggled with operational costs, due to the currency devaluations, especially affecting the ability to secure oxygen and medical supplies which are imported and priced in hard currency [34]. Some hospitals have had to operate at 50% capacity or less or resort to complete closure. Access to prevention-focused primary healthcare, including routine immunisation, has decreased, and there are large gaps in critical supply chains [15]. Fuel and electricity are a particular problem, with hospitals struggling to run generators and provide power for healthcare equipment [35]. Many health workers and skilled professionals have left the country, putting a huge strain on those remaining [36]. A shift in demand for health services from the private to the more affordable public sector has placed an additional strain on the already overstretched public hospitals that are grappling with decreasing incomes and increasing expenses.*

## 5. Deciding the Optimal Strategy for an Oxygen Ecosystem

The optimal oxygen ecosystem needs to take into consideration all the issues described above—the production and delivery to facilities, the system maintenance and quality control within facilities, data collection and monitoring, and the clinical use (Figure 2). The choice of the ecosystem depends on the local context such as existing infrastructure and resources, geography, economic climate, and available human, physical, and financial resources.

The majority of high- and upper-middle income countries use mostly LOX for historical reasons—PSA technologies are newer—in addition to the abundance of existing industries, expertise, and infrastructure that are able to maintain an LOX-based system. However, in Canada, PSA plants have been operational in 52 hospitals for over 30 years in parallel to the LOX system, and a study in 1999 found the system to be high-quality, with lower costs for oxygen and no patient care critical incidents [37]. In Peru, 175 oxygen PSA plants have been successfully installed nationwide [38].

A lack of sufficient oxygen production has been a chronic and critical problem for many low- and lower middle-income countries. During the COVID-19 pandemic, many countries developed large oxygen scale-up plans that predominantly used PSA-plant strategies, including Malawi, Uganda, Liberia, Ethiopia, Nigeria, and Vietnam [38]. Key principles in many of the plans are to ensure that the effective coverage of oxygen is increased and that the oxygen ecosystem is sustainable. In settings where much of the population cannot receive oxygen due to a lack of production and supply, increased supply is essential, and a technology mix may be appropriate.

As oxygen ecosystems are complex and are an essential part of any health system, it is recommended to have a National Oxygen Committee—a government-appointed body that is responsible for overseeing and coordinating the production, distribution, and use of medical oxygen in a country. The specific responsibilities of the committee can vary depending on the country but typically include establishing national standards, regulations, and policies, overseeing the distribution and use of medical oxygen, and ensuring a safe, effective, and sustainable oxygen ecosystem. In addition, the oxygen ecosystem should be embedded in the wider context of the health system. Engineering, clinical capacities, infrastructure, equipment, and supplies that benefit oxygen systems should also benefit the rest of the health system.

When deciding the way to run the oxygen ecosystem, failure tree analysis (FTA) can be useful. FTA is a structured method of identifying and analysing the potential causes and consequences of a failure or accident in a system, process, or equipment. The goal of FTA is to identify all possible failure modes, evaluate the likelihood of each failure mode, and determine the potential consequences of each failure mode. Economic evaluations of oxygen systems should use full life-cycle costs to include the total costs over the entire life span, from acquisition to retirement or disposal, taking into account not only the initial purchase price but also the costs of operating, maintaining, and disposing. Importantly, given oxygen costs are only 1-2% of the total budget for a small- or middle-sized hospital, other considerations than cost may be more important when deciding the form of oxygen production.

*Following the COVID-19 pandemic in Lebanon, the MOPH, UNICEF, and WHO have had concerns regarding the sustainability and resilience of the existing oxygen ecosystem in the country. Particular concerns have been around the cost and the overdependence on private LOX supplies, the increase in demand for oxygen due to a greater awareness of oxygen, and the use of high-flow oxygen. Plans have been developed for strengthening the oxygen ecosystem, including the extensive assessment that has formed the basis of this paper. Ten additional PSA plants are planned in public hospitals, while private hospitals have installed PSA plants for the provision of some of their baseline oxygen need. UNICEF has developed 18 recommendations for strengthening the oxygen ecosystem in Lebanon (Box 1). These include the establishment of a National Oxygen Committee, installation of an additional two PSA plants, strengthened systems for maintenance and electricity supply, increased production, procurement, and supply chain resilience, improved training and human resources, the use of data collection and regular information to guide the ecosystem, and integration of oxygen into the rest of the health system.*

## 6. Conclusions

Oxygen ecosystems in middle-income countries should be context appropriate and take into consideration the production of oxygen and delivery to facilities, the maintenance system within facilities, and the clinical use of oxygen. In Lebanon, eighteen recommendations for strengthening the oxygen ecosystem include the establishment of a National Oxygen Committee, installation of an additional two oxygen plants, strengthening systems for maintenance and electricity supply, increasing production, procurement, and supply chain resilience, improving training and human resources, and the use of data collection and regular information to guide the integration of oxygen into the rest of the health system.

## Figures and Tables

**Figure 1:** Comparison of LOX and PSA with reference to Lebanon. ^*∗*^Authors' estimates using calculations performed in the 2022-2023 assessment conducted by the government and UNICEF.

**Figure 2:** Oxygen ecosystem: four requirements for health impact. 1a: Establish policies such as national oxygen roadmaps and national oxygen committees to enable context-appropriate planning of the oxygen ecosystem. 1b: Gather information about the need, access, and provision of oxygen to guide policy and planning. 2a: Produce sufficient oxygen for the needs of the population. 2b: Maintain safe, efficient, and sustainable oxygen production and integrate the oxygen ecosystem with the rest of the health system. 3a: Establish reliable oxygen delivery systems within health facilities. 3b: Maintain safe, efficient, continuous, and sustainable oxygen delivery systems in health facilities and integrate with the rest of the facility. 4a: Treat patients with oxygen effectively and appropriately. 4b: Treat oxygen-requiring patients with the other essential care they need. 4c: Ensure the clinical use of oxygen is sustainable and integrated with other care provision.

**Algorithm 1:** Recommendations for strengthening the oxygen ecosystem in Lebanon.

## Data Availability

Data sharing is not applicable to this article as no datasets were generated or analysed during the current study.

## Abbreviations

GDP: Gross domestic product
FTA: Failure tree analysis
LOX: Liquid oxygen
MOPH: Ministry of Public Health
PSA: Pressure swing adsorption
VSA: Vacuum swing adsorption.
